# Protective Effects of Platycodin D3 on Airway Remodeling and Inflammation via Modulating MAPK/NF-*κ*B Signaling Pathway in Asthma Mice

**DOI:** 10.1155/2022/1612829

**Published:** 2022-08-10

**Authors:** Feng Peng, Fengchun Xiao, Long Lin

**Affiliations:** ^1^Department of Pediatrics, Affiliated Hangzhou Chest Hospital, Zhejiang University School of Medicine, Hangzhou 310003, China; ^2^Department of Pediatrics, Zhejiang Hospital of Integrated Traditional Chinese and Western Medicine, Hangzhou 310003, China; ^3^Department of Pathology, The First Affiliated Hospital of Zhejiang Chinese Medical University, Hangzhou 310016, China

## Abstract

**Background:**

Asthma is a disease with airway hyperresponsive and airway inflammation. Platycodin D is a triterpenoid saponin extracted from *Platycodon grandiflorus* root, which has various pharmacological activities. The study mainly explored the effects of platycodin D3 (PD_3_) in airway remodeling and inflammation of asthma.

**Methods:**

The ovalbumin (OVA)-induced asthma mice were given PD3 (20 mg/kg, 40 mg/kg, and 80 mg/kg) in different groups. The asthma mice administrated with dexamethasone (DXM) were enrolled as the positive control group, and the normal control mice and asthma model mice separately received the same volume of saline. Mouse airway lung dynamic compliance (Cdyn) and total airway resistance (RL) were measured by the EMKA animal lung function analysis system. The inflammation factor levels were estimated by ELISA. Histopathological changes were tested by HE and PAS staining. The protein and phosphorylation levels of NF-*κ*Bp65, p38, ERK1/2, and JNK1/2 were detected by Western blot.

**Results:**

In asthmatic mice, PD3 enhanced the airway Cdyn and decreased RL to improve the airway hyperreactivity and alleviated the pathological injury of lung tissues. In addition, PD3 could reduce the infiltration of inflammatory cells in BALF and suppress the levels of eotaxin, IL-4, IL-5, IL-13, IFN-*γ*, and IgE. Furthermore, PD3 treatment inhibited the phosphorylation of NF-*κ*Bp65, p38, ERK1/2, and JNK1/2 proteins in asthma mice.

**Conclusion:**

PD3 treatment alleviated the airway remodeling and inflammation in asthmatic mice, which might be related to downregulating the phosphorylated proteins in the MAPK/NF-*κ*B signaling pathway.

## 1. Introduction

Asthma is an airway disease characterized by chronic inflammation in the airways [1]. The clinical manifestations are episodic wheezing or coughing [2]. Asthma morbidity and mortality are rising globally [3]. Its pathological features are mainly airway hyperresponsiveness (AHR), airway chronic inflammation, and gradually airway remodeling [4]. Relevant research had shown that airway remodeling was an important reason that made asthma difficult to cure [5]. Glucocorticoids, the most effective anti-inflammatory drugs at present, were widely used clinically as first-line antiasthma drugs [6]. However, O'Byrne et al. found that glucocorticoids had great individual differences in inhibiting airway remodeling, and if they were used for a long time, adverse reactions such as metabolic disorders and growth inhibition would occur [7]. Therefore, there is still a need to continuously explore new antiasthma drugs.

NF-*κ*B played a vital part in the inflammation, immune responses, and tumor [8]. Moreover, research studies had shown that NF-*κ*B could change the levels of various inflammatory factors [9, 10]. NF-*κ*B had been found to be activated in asthma patients and animal models, and inhibition of NF-*κ*B could prevent the occurrence of asthma [11]. The MAPK pathway existed widely and regulated many biological processes, such as cell growth and proliferation [12]. MAPK had been seen as a key signaling molecule that promoted inflammation [13]. Yuan et al. found that JAX2 prevented bronchial asthma by inhibiting MAPK/NF-*κ*B inflammatory signaling [14]. Therefore, NF-*κ*B and MAPK had become molecular targets for asthma therapy [15].

*Platycodon grandiflorus* (Jacq.) A.DC is a traditional Chinese medicinal material and food and has the functions of dispersing the lung, soothing the throat, expectorating phlegm, and relieving cough [16]. Platycodin D (PD), an effective triterpene saponin isolated from the root of *Platycodon grandiflorus*, had been reported to have anti-inflammatory, antitumor, and antioxidative effects [17]. Among them, the common triterpenoid saponins were platycodin D3 (PD3) and platycodin A [18]. In recent years, the pharmacological effects of PD in regulating Th1/Th2 immune balance, anti-inflammatory and expectorant, and antitumor had attracted the attention of researchers [19]. It has been reported that PD had a vital therapeutic effect on allergic asthma model mice, reducing airway resistance and eosinophils and inflammatory factors by inhibiting NF-*κ*B [20]. It has been recently reported that natural herbal saponins could inhibit ovalbumin-induced levels of the inflammatory factor IL-17A in mice, thereby reducing the inflammatory symptoms of asthma [21]. Sung et al. found that saponin extract had a certain alleviation effect on ovalbumin-induced airway inflammation and airway remodeling in the asthma model [22]. Fu et al. found that PD protected against acetaminophen-induced hepatotoxicity by regulating the MAPK pathway in mouse hepatocytes [23]. Besides, it was showed that PD and PD3 increased airway mucin secretion to resolve airway phlegm in the animal model [24]. However, the molecular mechanism of PD3 in asthma remains unclear.

The study explored the protective effect of PD3 on airway remodeling and inflammation in asthmatic mice by regulating the MAPK/NF-*κ*B signaling pathway.

## 2. Materials and Methods

### 2.1. Asthma Mice Model Establishment and Treatment

The six-week-old male BALB/*c* mice (6–8 w, 18–20 g) were brought from Shanghai Lingchang Biotech Co., Ltd. (Shanghai, China). They were reared under SPF conditions and had free access to food and water. They were randomly divided into 6 groups (*n* = 6): one group mice were ranked as the control group and were given normal saline injection and other five groups received the ovalbumin (OVA) (^#^S7951, sigma) medium (0.5 ml/each) with aluminum hydroxide for eight weeks. In addition, the asthma mice in the PD3 (^#^67884-03-1, eBiochemicals) group were treated with PD3 at 20, 40, and 80 mg/kg/d, respectively; the asthma mice in the dexamethasone (DXM) (^#^ID0170, Solarbio) group received DXM 0.5 mg/kg/d.

### 2.2. AHR Measurement

After final drug treatment, all the mice were put in the EMKA animal lung function analysis system and successively inhaled saline, methacholine (^#^PHR1943, sigma) at different concentrations (0.0625, 0.125, 0.25, 0.5, 1.0, and 2.0 mg/ml). Besides, the airway lung dynamic compliance (Cdyn) and total airway resistance (RL) in each mouse were recorded and analyzed.

### 2.3. BALF Was Collected and Cell Counted

Mice were euthanized by CO_2_. Then, the lungs were washed with cold PBS. Afterwards, the BALF samples were centrifuged and then suspended in PBS, and the total number of cells was counted. Later cell medium was centrifuged, and the inflammatory cell counts were analyzed with Wright–Giemsa staining (^#^G1020, Solarbio).

### 2.4. ELISA Assay

The levels of IL-4, IL-5, IL-13, IFN-*γ*, and chemokine (eotaxin) in BALF and the total serum IgE were analyzed by IL-4 ELISA kits (^#^70-EK204/2–96, MultiSciences), IL-5 ELISA kits (^#^70-EK205-96, MultiSciences), IL-13 ELISA kits (^#^70-EK213/2–96, MultiSciences), IFN-*γ* ELISA kits (^#^70-EK280/3–96, MultiSciences), Eotaxin ELISA kits (^#^70-EK2130/2–96, MultiSciences), and IgE ELISA kits (^#^6370, Amercian Diagnostica Inc.).

### 2.5. HE and PAS Staining

The lung tissue was fixed with paraformaldehyde and embedded in paraffin. Then sectioned into 4 *μ*m thick pieces, the sections received ethanol dehydration of different concentrations. Lung tissue was stained by HE staining (^#^G1120, Solarbio) and periodic acid Schiff (PAS) staining (^#^ab150680, Abcam), and its pathological changes were observed under a microscope.

### 2.6. Western Blot

First, the total protein was collected and the concentration was detected by the BCA protein kit (Solarbio, pc0020). The PVDF membrane was blocked by a blocking solution, and the membrane was put into the primary antibodies: NF-*κ*Bp65 antibody (^#^ab16502, Abcam), pNF-*κ*Bp65 antibody (^#^ab86299, Abcam), p38 antibody (^#^ab31828, Abcam), p-p38 antibody (^#^ab47363, Abcam), ERK1/2 antibody (^#^ab17942, Abcam), pERK1/2 antibody (^#^ab214362, Abcam), JNK1/2 antibody (^#^ab112501, Abcam), and pJNK1/2 antibody (^#^ab131499, Abcam) and then incubated overnight. Afterwards, the anti-mouse IgG antibody was added. The protein bands were detected by ECL chemiluminescence instrument and chemi-capture software. Finally, the proteins' gray intensity was analyzed with ImageJ software.

### 2.7. Statistical Analysis

SPSS software (16.0, IBM, USA) was used for data analysis. Student's *t*-test was used for two groups comparison. One-way ANOAY followed by the Tukey test was utilized for multiple groups comparison if it was normally distributed. The Kruskal–Wallis H test was utilized if it was not normally distributed. All data were described as mean ± standard deviation (SD). *P* < 0.05 suggested that the difference was statistically significant.

## 3. Results

### 3.1. PD3 Treatment Alleviated the AHR

The effects of PD3 on AHR were evaluated with airway Cdyn and RL. The results showed that the airway Cdyn reduced after inhaling different concentrations of methacholine (0.0625, 0.125, 0.25, 0.5, 1.0, and 2.0 mg/ml), whilst the airway RL increased. However, giving different concentrations of PD3 (20, 40, and 80 mg/kg/d) enhanced the airway Cdyn and alleviated the airway RL (Figure 1).

### 3.2. PD3 Treatment Reduced the Airway Inflammatory Cell Counts

The airway inflammatory cell counts were detected in the BALF. The results in Figure 2 showed that, compared with the control group, the total number of inflammatory cells, eosinophils, macrophages, lymphocytes, and neutrophils increased in the asthma group. Administration of different concentrations of PD3 (20, 40, and 80 mg/kg/d) treatment significantly reduced the total number of inflammatory cells, eosinophils, macrophages, lymphocytes, and neutrophils, further reducing airway inflammation.

### 3.3. PD3 Treatment Reduced the Levels of Airway Inflammatory Cytokines and IgE

The effects of PD3 on the levels of IL-4, IL-5, IL-13, IFN-*γ*, eotaxin, and IgE in BALF were detected by ELISA, and the results are shown in Figure 3. The levels of IL-4, IL-5, IL-13, IFN-*γ*, eotaxin, and IgE in the asthma group were significantly higher than those in the control group. However, treatment with different concentrations of PD3 (20, 40, and 80 mg/kg/d) significantly reduced the levels of airway inflammatory factors and IgE.

### 3.4. PD3 Treatment Alleviated Airway Pathological Changes

The pathological changes of the lung tissue were observed by HE staining and PAS staining. The results of HE staining are shown in Figure 4(a), and inflammatory cell infiltrations were found in the airway tissue in the asthma group. However, the inflammatory cell infiltration significantly reduced after treatment with different concentrations of PD3 (20, 40, and 80 mg/kg/d).

Moreover, the results of PAS staining are shown in Figure 4(b). It was found that in the lung tissue of asthmatic mice were characterized mucus hypersecretion and goblet cells hyperplasia. However, giving different concentrations of PD3 (20, 40, and 80 mg/kg/d), the secretion of mucus and goblet cells hyperplasia in the lung tissue decreased, and the pathological characteristics were alleviated.

### 3.5. PD3 Treatment Reduced the Expression of Proteins Associated with the MAPK/NF-*κ*b Signaling Pathway

The expressions of pNF-*κ*Bp65, p-p38, pERK1/2, and pJNK1/2 protein in the lung tissue were detected by Western blot and the results are shown in Figure 5. The expressions of pNF-*κ*Bp65, p-p38, pERK1/2, and pJNK1/2 in the asthma group were higher than those in the control group. The expressions of pNF-*κ*Bp65, p-p38, pERK1/2, and pJNK1/2 all decreased after giving different concentrations of PD3. However, further observation found that the expressions of pNF-*κ*Bp65, p-p38, pERK1/2, and pJNK1/2 in the PD3 (20 mg/kg) group protein did not decrease significantly, and the expressions of pNF-*κ*Bp65, p-p38, pERK1/2, and pJNK1/2 significantly reduced in the PD3 (40 mg/kg, 80 mg/kg) group.

## 4. Discussion

Asthma is a common and frequent chronic respiratory disease [25]. PD3 is a traditional Chinese medicine with anti-inflammatory and immune effects. Moreover, PD3 has been reported to regulate airway mucin secretion [26]. Our study found that PD3 could alleviate the airway remodeling and inflammation in asthmatic mice, which might be achieved by regulating the MAPK/NF-*κ*B pathway.

This study found that PD3 treatment enhanced airway Cdyn and alleviated airway RL, which was similar to the study by Shin et al. that PD3 improved airway function and prevented airway inflammation [24]. In addition, we found that the inflammatory cells and the levels of inflammatory factors in asthmatic mice were higher. However, they were reversed after giving different concentrations of PD3 treatment, which was concordant with the results of Lee et al.; they found that PD inhibited the inflammatory factors in OVA asthmatic mice [27]. Lee et al.'s study also proved that *Platycodon grandiflorus* fermented extract could reduce the total number of cells and eosinophils in guinea pig BALF and reduce the levels of inflammatory factors [28]. This study further found that PD3 could improve the pathological changes of the lung tissue in asthmatic mice and had a protective effect on airway remodeling and inflammation. The results of this study were consisted with those of previous studies, which showed that *Platycodon grandiflorus* extract could inhibit the infiltration of mucous inflammatory cells [29].

In addition, studies have found that MAPK/NF-*κ*B signaling acted as an inflammatory promoter and could control asthmatic airway responses via regulating the MAPK/NF-*κ*B pathway [30, 31], as well as inhibit lung inflammation in asthmatic mice [32]. Previous studies had found that airway remodeling could be improved through regulating the MAPK/NF-*κ*B pathway [33, 34]. Moreover, Jang et al. found that platycodin had an inhibitory effect on cellular inflammatory factors by the NF-*κ*B/MAPK pathway [35]. In this study, the expressions of phosphorylation NF-*κ*Bp65, p38, ERK1/2, and JNK1/2 elevated in asthmatic mice. However, NF-*κ*B/MAPK pathway-related protein levels were reversed after administration of PD3. Wang et al. found that platycodin D alleviated expressions of the phosphorylated proteins in NF-*κ*B/MAPK signaling pathway which contributed to the inhibition of the airway inflammation [36].

Hence, the study found that PD3 could suppress airway inflammation by relieving the expression of phosphorylated proteins in the NF-*κ*B/MAPK signaling pathway. However, this study also has certain limitations. The mechanism for action of PD3 against asthma has not been fully confirmed and needs to be further explored.

## 5. Conclusion

Taken together, PD3 has protective effects on airway remodeling and inflammation in asthmatic mice by downregulating the phosphorylated proteins of the NF-*κ*B/MAPK signaling pathway.

## Figures and Tables

**Figure 1:** PD_3_ treatment enhanced Cdyn and reduced RL in a dose-dependent manner. (a) Airway dynamic compliance (Cdyn). (b) Lung resistance (RL) in the asthma mice model. PD3, platycodin D3. Data were expressed as mean ± SD, *n* = 3. Compared with the control group, ^★^*P* < 0.05, ^★★^*P* < 0.01. Compared with the asthma group, ^#^*P* < 0.05, ^##^*P* < 0.01.

**Figure 2:** PD3 treatment reduced total inflammatory cells (a), total eosinophils (b), macrophages (c), lymphocytes (d), and neutrophils (e) in BALF. PD3, platycodin D3. Data were expressed as mean ± SD, *n* = 3. Compared with the control group, ^★^*P* < 0.05, ^★★^*P* < 0.01. Compared with the asthma group, ^#^*P* < 0.05, ^##^*P* < 0.01.

**Figure 3:** PD3 treatment reduced (a) Eotaxin, (b) IL-4 , (c) IL-5, (d) IL-13 (e) IFN-*γ*, (f) serum OVA-specific IgE levels in BALF. PD3: Platycodin D3. Data were expressed as mean ± SD, *n* = 6. Compared with the control group, ^★^*P* < 0.05, ^★★^*P* < 0.01; Compared with the Asthma group ^#^*P* < 0.05, ^##^*P* < 0.01.

**Figure 4:** (a) HE staining of asthma mice lung tissues, PD_3_ treatment alleviated airway pathological lesion. Blue arrows pointed the inflammatory cells immersed in the lung tissues. The 200x scale bar was 100 *μ*m; the 400x scale bar was 50 *μ*m. (b) AB-PAS staining of asthma mice lung tissues, PD_3_ treatment alleviated airway mucus secretion and goblet cells hyperplasia. The 200x scale bar was 100 *μ*m; the 400x scale bar was 50 *μ*m. PD3, platycodin D3.

**Figure 5:** PD3 treatment reduced the expression of proteins associated with the MAPK/NF-*κ*B signaling pathway. (a) Bands of NF-*κ*Bp65 and p-NF-*κ*Bp65, p38 and p-p38, ERK1/2 and p-ERK1/2, and JNK1/2 and p-JNK1/2 proteins. PD3 treatment reduced the expression levels of NF-*κ*Bp65 and p-NF-*κ*Bp65 (b), p38 and p-p38 (c), ERK1/2 and p-ERK1/2 (d), and JNK1/2 and p-JNK1/2 (e) proteins. PD3, platycodin D3. Data were expressed as mean ± SD, *n* = 3. Compared with the control group, ^★^*P* < 0.05, ^★★^*P* < 0.01; compared with the asthma group, ^#^*P* < 0.05, ^##^*P* < 0.01.

## Data Availability

The data used to support this study are included within the article.

## Additional Points

Platycodin D3 reduces inflammatory cells and cytokines to improve pathological injury of lung tissues in asthmatic mice. Platycodin D3 inhibits phosphorylation of the MAPK/NF-*κ*B pathway in asthmatic mice.
